The article "S100A8 Contributes to Drug Resistance by Promoting Autophagy in Leukemia Cells" was retracted in 2020. Reasons: manipulated images; errors in the images; duplicated images; concerns about the images.

# S100A8 Contributes to Drug Resistance by Promoting Autophagy in Leukemia Cells

**DOI:** 10.1371/journal.pone.0097242

**Published:** 2014-05-12

**Authors:** Minghua Yang, Pei Zeng, Rui Kang, Yan Yu, Liangchun Yang, Daolin Tang, Lizhi Cao

**Affiliations:** 1 Department of Pediatrics, Xiangya Hospital, Central South University, Changsha Hunan, China; 2 Department of Infectious Diseases, Xiangya Hospital, Central South University, Changsha, Hunan, China; 3 Department of Surgery, University of Pittsburgh Cancer Institute, Pittsburgh, Pennsylvania, United States of America; University of Manitoba, Canada

## Abstract

Autophagy is a double-edged sword in tumorigenesis and plays an important role in the resistance of cancer cells to chemotherapy. S100A8 is a member of the S100 calcium-binding protein family and plays an important role in the drug resistance of leukemia cells, with the mechanisms largely unknown. Here we report that S100A8 contributes to drug resistance in leukemia by promoting autophagy. S100A8 level was elevated in drug resistance leukemia cell lines relative to the nondrug resistant cell lines. Adriamycin and vincristine increased S100A8 in human leukemia cells, accompanied with upregulation of autophagy. RNA interference-mediated knockdown of S100A8 restored the chemosensitivity of leukemia cells, while overexpression of S100A8 enhanced drug resistance and increased autophagy. S100A8 physically interacted with the autophagy regulator BECN1 and was required for the formation of the BECN1-PI3KC3 complex. In addition, interaction between S100A8 and BECN1 relied upon the autophagic complex ULK1-mAtg13. Furthermore, we discovered that exogenous S100A8 induced autophagy, and RAGE was involved in exogenous S100A8-regulated autophagy. Our data demonstrated that S100A8 is involved in the development of chemoresistance in leukemia cells by regulating autophagy, and suggest that S100A8 may be a novel target for improving leukemia therapy.

## Introduction

Autophagy is a catabolic process involving the degradation of intracellular aggregated or misfolded proteins, and damaged organelles through lysosomal machinery in response to stress or starvation [1], [2]. Deregulation of autophagy is implicated in several human diseases including cancers. Depending on the type of tumor and stage of disease, autophagy induces both tumor cell survival and death during the initiation, progression, maturation and maintenance of cancer [3].

It has been well documented that autophagy plays an important role in the resistance of cancer cells to chemotherapy [4]. Consequently, pharmacological inhibition of autophagy enhances chemotherapeutic drug-induced cytotoxicity and apoptosis in leukemia cells [4]–[6]. We recently found that damage associated molecular pattern molecules (DAMPs) such as high mobility group box 1 (HMGB1) contribute to chemotherapy resistance though upregulating autophagy in leukemia [7]. S100A8 (also designated MRP8 or calgranulin A) is a member of DAMPs, differentially expressed in a wide variety of cell types and abundant in myeloid cells [8], [9]. S100A8 is involved in the progression of various cancers, including leukemia, and induces cell death by functional linkage with Bcl-2 family members [10]–[14]. We previously found that the expression level of S100A8 correlates with poor clinical outcomes in childhood acute myeloblastic leukemia (AML). Accordingly, knockdown of S100A8 by siRNA-treated myeloid leukemia cells showed sensitization to arsenic trioxide, accompanied with the attenuation of autophagy and disassociation of the BECN1-Bcl-2 complex [14]. The data suggest that S100A8 contributes to chemoresistance *via* regulating the autophagy in leukemia.

In this study, we found that S100A8 enhances drug resistance by upregulating autophagy through promoting the formation of BECN1-PI3KC3 [PI3KC3, phosphatidylinositol 3-kinase class 3] complex, providing a novel potential target for the treatment of leukemia.

## Materials and Methods

### Antibodies and reagents

The antibodies against S100A8 and p62 were obtained from Santa Cruz Biotechnology (Sana Cruz, CA, USA). The antibodies to Actin, BECN1, PI3KC3, C-PARP, ULK1, Bcl-2 and P-ULK1 were from Cell Signaling Technology (Boston, MA, USA). The antibodies to LC3 and TLR-4 were purchased from Abcam (Cambridge, MA, USA). Anti-Atg7 antibody was from Novus (Denver-Littleton, CO, USA). Vincristine (VCR), adriamycin (ADM), rotenone (Rot), thenoyltrifluoroacetone (TTFA), antimycin A (AA), E64D, anti-RAGE antibody and pepstatin were from Sigma (Milpitas, CA, USA). Full-length human S100A8 cDNA (pLPCX-S100A8) was a gift from Dr. RW Stam (Erasmus Medical Center/Sophia Children's Hospital, Netherlands). FITC-Annexin V Apoptosis Detection kit and the Nuclear and Cytoplasmic Protein Extraction kit were purchased form Beyotime Institute of Biotechnology (Beijing, China). S100A8 protein was obtained from Novus Biologicals. Contaminating LPS was removed by Triton X-114 extraction. LPS content was always below 0.5 ng/mg protein, which did not cause an effect in our assays.

### Cell culture

The human leukemia cell lines, K562 (chronic myeloid leukemia cells), HL-60 (acute myeloid leukemia cells), MV-4-11 (biphenotypic B myelomonocytic leukemia cells), Jurkat (T-cell acute lymphoblastic leukemia cells), and K562/A02 (multidrug resistance K562) were from the American Type Culture Collection; HL-60/ADR (multidrug resistance HL-60) was from the Institute of Hematology & Blood Diseases Hospital of Chinese Academy of Medical Sciences & Peking Union Medical College. Cells were cultured in RPMI-1640 medium supplemented with 10% heat-inactivated FBS and 2 mM glutamine in a humidified incubator with 5% CO2 and 95% air.

### Cell viability assay

Cell viability was assessed by MTT assay. Briefly, leukemia cells were seeded in 96-well plates (4000 cells/well) the day before treatment. Following treatment with ADR for 72 h, 25 µL MTT [3-(4,5-dimethylthiazol–2-yl)- 2,5-diphenyltetrazolium bromide; Sigma] was added to each well and incubated for 3.5 h, followed by the addition of 100 µL of N,Ndimethylformamide (D4551; Sigma). The plates were left at room temperature overnight to allow complete lysis of the cells, and read at 450 nm the following day. Half-maximal inhibitory concentration (IC50) was calculated using MS Excel, as previously described [15].

### Western blot analysis

Cell lysates were prepared with cell lysis buffer [20 mmol/L Tris-HCl, pH 7.5; 150 mmol/L NaCl; 1 mmol/L Na2EDTA; 1 mmol/L EGTA; 1% Triton; 2.5 mmol/L sodium pyrophosphate; 1 mmol/L b-glycerophosphate; 1 mmol/L Na3VO4; 1 mg/mL leupeptin; 1 mmol/L phenylmethylsulfonylfluoride (PMSF); and 1 mmol/L PMSF], and cleared by centrifugation. Total protein concentration was determined with the bicinchoninic acid assay Kit (Bio-Rad). Proteins were resolved on a denaturing 10% SDS-PAGE gel and subsequently transferred to polyvinylidene fluoride membranes *via* semidry transfer. The membrane was blocked with 5% dried milk or 3% bovine serum albumin in Tris-buffered saline and Tween 20 (10 mmol/L Tris, pH 7.5; 100 mmol/L NaCl; and 0.1% Tween20), incubated with primary antibodies, and then with horseradish peroxidase–conjugated secondary antibodies. The signals were visualized by enhanced chemiluminescence.

### Quantitative real-time PCR

Total RNA was extracted using TRIzol (Invitrogen, USA) according to the manufacturer's instructions. Reverse transcription (RT) was performed with 2 µg of total RNA with HiFi-MMLV Enzyme Mix (CWbio, China). Twenty ng cDNA was subjected to real-time quantitative PCR (TaqMan probes) for the evaluation of the relative S100A8 mRNA, with beta actin as an internal control with gene specific primers and fluorogenic probes (S100A8: forward primer 5′- CCTAACCGCTATAAAAAGGAG -3′, reverse primer 5′- ATGATGCCCACGGACTTGCC -3, probe 5′ FAM-CCTCTCAGCCCTGCATGTCTCTT -TAMRA 3′; ACTB: forward primer 5′- GGCACCCAGCACAATGAAGA-3, reverse primer 5′-CGTCATACTCCTGCTTGCTG-3′, probe 5′FAM-CTGGAAGGTGGACAGCGAGGC-TAMRA 3′.) in an LightCycler 480 **System** (Roche). Quantification was determined by the standard curve and 2-ΔΔCt methods [15].

### Immunoprecipitation analysis

Cells were lysed at 4°C in ice-cold radioimmunoprecipitation assay lysis buffer (Millipore, Billerica, MA, USA). Cell lysates were cleared by a brief centrifugation (12,000 g, 10 min). Protein concentration in the supernatant was determined by bicinchoninic acid assay. Before immunoprecipitation, equal amounts of proteins were pre-cleared with Protein A or protein G agarose/sepharose (Millipore) at 4°C for 3 h and subsequently incubated with various irrelevant immunoglobulin-G or specific antibodies (5 µg/ml) in the presence of protein A or G agarose/sepharose beads for 2 h or overnight at 4°C with gently shaking. Following incubation, agarose/sepharose beads were washed extensively with phosphate buffered saline. Proteins were eluted by boiling in 2×SDS sample buffer before SDS–polyacrylamide gel electrophoresis and immunoblot analysis, as previously described [15], [16].

### Gene transfection and RNAi

Cells were transfected with S100A8 pLPCX constructs by square-pulse electroporation at 600 V for 2 msec and cultured under selection of neomycin (1 mg/ml; Gibco BRL, USA) and puromycin (10 mg/ml; Sigma) in order to obtain a pure population of transfected cells [13]. Lipofectamine 2000 Transfection Reagent (Invitrogen) was used to transfect S100A8-shRNA, BECN1-shRNA, PI3KC3-shRNA, ULK1-shRNA, RAGE-shRNA, TLR4-shRNA and Atg7 shRNA (Sigma) [16]. As a control experiment, another S100A8-shRNA was obtained from Gene Pharma (Shanghai, China).

### Apoptosis assays

Apoptosis was assessed using the FITC Annexin V Apoptosis Detection kit, which involves staining cells with Annexin V-FITC (a phospholipid-binding protein that binds to disrupted cell membranes) in combination with PI (a vital dye that binds to DNA penetrating into apoptotic cells). Flow cytometric analysis (FACS) was performed to determine the percentage of apoptotic cells (Annexin V^+^/PI).

### Electron microscopy

Leukemia cells were collected and fixed in 2.5% glutaraldehyde for at least 3 h. Then cells were treated with 2% paraformaldehyde at room temperature for 60 min, 0.1% glutaraldehyde in 0.1 M sodium cacodylate for 2 h, post-fixed with 1% OsO4 for 1.5 h, dehydrated with graded acetone, and embedded in Quetol 812. Ultrathin sections were observed using a Hitachi H7500 electron microscope (Tokyo, Japan) [17].

### Immunofluorescence and confocal microscopy

Cells were collected, fixed and permeabilized with 0.3% triton X-100 for 10 min, incubated with anti-LC3 for 1 h and then FITC-conjugated Anti-LC3A/B antibody (Abcam, ab58610) for 1 h at room temperature. Cell nuclei were stained using ProLong Gold Antifade Reagent with DAPI (Life Technologies). Samples were examined under an Olympus FV1000 confocal microscope. For evaluating tandem fluorescent LC3 puncta, cells were washed with PBS, fixed with 4% paraformaldehyde, mounted with DAPI and viewed under a confocal microscope [17].

### Autophagy assays

To analyze autophagic flux, we monitored the formation of autophagic vesicles by the mRFP–GFP–LC3 method (Invitrogen). Due to the quenching of GFP in the acidic lysosomal environment [17], we could distinguish the autophagosomes and autolysosomes through detecting both mRFP and GFP signals, followed by only the mRFP signal. K562 cells were transfected with mRFP-GFP-LC3 expressing pLenti6 lentivirus (Nanjing Mergene Life Science, Nanjing, China). Autophagic flux was determined by evaluating the punctuated pattern of GFP and mRFP (punctae/cell were counted). Fluorescence was analyed on an Olympus (Aartselaar, Belgium) cell imaging station using Cell M software. The protein levels of LC3 and p62 were determined by Western blotting. Transmission electron microscopic (TEM) assessment of autophagosomes-like structures was performed as previously described [7].

### Statistical analysis

All experiments were performed in at least triplicates per group, and data are reported as mean±SEM, unless otherwise indicated. Data were analyzed by 2-tailed Student *t*-test or ANOVA least significant difference test, and P<0.05 was considered significant.

## Results

### S100A8 was overexpressed in drug resistance leukemia cells and anticancer agents increased S100A8 expression in leukemia cells

S100A8 was differentially expressed in different cell lines, with relatively low S100A8 in Jurkat cells. We found that S100A8 protein was significantly increased in the drug resistance leukemia cell line K562/A02, relative to the nondrug resistant cell line K562 (Fig. 1A). Elevated S100A8 protein level was also observed in the drug resistance HL-60/ADR cells compared to HL-60 cells (Fig. 1A). Furthermore, there were relatively high levels of S100A8 mRNAs in HL-60, K562 and MV4-11 cells in comparison to Jurkat cells (Fig. 1B), and significantly increased S100A8 mRNAs in K562/A02 and HL-60/ADR compared with K562 and HL-60, respectively (Fig. 1C). These results showed that drug-resistant leukemia cells overexpress S100A8.

**Figure 1:** S100A8 was elevated in drug resistance leukemia cells and chemotherapy agents induced S100A8 expression in leukemia cells. (**A**) Protein level of S100A8 was analyzed by Western blotting in Jurkat, HL-60, K562 and MV4-11 cells (n = 3, ^*^ *P*<0.05). (**B and C**) S100A8 mRNA level in leukemia cells was analyzed by real time RT-PCR (n = 3, ^*^ *P*<0.05 versus Jurkat cells in **B** and ^*^ *P*<0.05 versus HL-60 or K562 in **C**, Jurkat group set as 1). (**D**) Basal LC3-I/II level was analyzed by Western blotting in leukemia cells (n = 3, ^*^ *P*<0.05 *versus* Jurkat cells ). (**E and F**) IC50 levels of adriamycin (ADR) in Jurkat, K562, HL-60, MV-4-11, K562/A02, and HL-60/ADR cells (n = 3, ^*^ *P*<0.05 versus Jurkat cells in **E**, ^*^ *P*<0.05 versus HL-60 or K562 in **F**). (**G**) Jurkat, HL-60, K562 and MV4-11 cells were treated with ADR (1 µg/ml), VCR (1 µg/ml) or As2O3 (5 µM) for 24 hours and S100A8 protein level was analyzed by Western blotting (n = 3, *P<0.05 vs. UT, untreated group). AU, arbitrary unit. (**H**) Jurkat, HL-60, K562 and MV4-11 cells were treated with ADR (1 µg/ml), vincristine (VCR, 1 µg/ml) or arsenic trioxide (As2O3, 5 µM) for 24 hours and S100A8 mRNA level was analyzed by real time RT-PCR (n = 3, *P<0.05 versus control group, control group set as 1).

At the same time, we found the basal authophagy level in the drug resistant leukemia cells was higher compared to the non-drug resistant cell lines. We evaluated basal authophagy in leukaemia cells and compared the levels of autophagy with S100A8 expression. Basal authophagy in leukaemia cells was low. Moreover, we found there were no significant difference in levels of LC3-II/LC-I in HL-60, K562 and MV4-11 cells in comparison to Jurkat cells. However, the authophagy level were increased in K562/A02 relative to K562, and HL-60/ADR compared to HL-60 (Fig. 1D).

To explore the functions of S100A8 in drug resistance, we next analyzed the relationship between the IC50 of adriamycin and the expression level of S100A8. Increased expression of S100A8 was correlated with higher IC50 of adriamycin (Fig. 1E). Overexpression of S100A8 in K562/A02 and HL-60/ADR cells was coincident with dramatic increase in IC50 of adriamycin (Fig. 1F), indicating that S100A8 plays an important role in the drug resistance of leukemia cells.

It was reported that chemotherapeutic drugs induce S100A8 in the supernatants of cell cultures [14]. To further determine the potential role of S100A8 in leukemia in response to chemotherapy, we quantified S100A8 of leukemia cells following treatment with vincristine (VCR, 1 µg/ml), adriamycin (ADR, 1 µg/ml), and arsenic trioxide (As2O3, 5 µM), which are widely used for the treatment of hematological malignancies. Treatment of K562, HL-60, Jurkat and MV4-11 cells with VCR, ADR and As2O3 for 24 h led to significant upregulation of S100A8 protein (Fig. 1G) and mRNA (Fig. 1H).

### Suppression of S100A8 rescued the chemotherapy sensitivity in drug resistance leukemia cells

To evaluate whether overexpression of S100A8 results in drug resistance, we knocked down S100A8 by shRNA in HL60/ADR and K562/A02. S100A8 shRNA transfection led to a significant decrease of both S100A8 protein and mRNA in these cells (Fig. 2A). Knockdown of S100A8 significantly sensitized these cells to adriamycin and Vincristine (Fig. 2B), accompanied with high levels of apoptotic cell death (Fig. 2C) and an increase in cleaved PARP1 (Fig. 2D). Moreover, S100A8 knockdown increased the activation of the proapoptotic protein caspase-3 by both adriamycin and Vincristine, which was abolished by addition of the pan-caspase inhibitor Z-VAD-FMK (Fig. 2E). In addition, knockdown of S100A8 in HL60/ADR cells by another S100A8 shRNA from Gene Pharma also increased the sensitivity to DRN- and VCR-induced suppression of cell proliferation and apoptosis (Fig. 2F). These data demonstrated that S100A8 increased the resistance of leukemia cells to cytotoxic agents and knockdown of S100A8 restored the sensitivity of K562/A02 and HL60/ADR cells to adriamycin and vincristine.

**Figure 2:** Suppression of S100A8 sensitized drug resistance leukemia cells to chemotherapy. **(A)** HL60/ADR and K562/A02 cells were transfected with control shRNA or S100A8 shRNA for 48 hours. Protein and mRNA level of S100A8 was assayed by Western blot and real time RT-PCR, respectively. (**B**) HL60/ADR and K562/A02 cells were transfected with control shRNA or S100A8 shRNA for 48 hours, then treated with adriamycin (ADR) and vincristine (VCR) for an additional 24 hours. Cell viability was analyzed by MTT. (**C and D**) HL60/ADR and K562/A02 cells were transfected with control shRNA or S100A8 shRNA for 48 hours, treated with ADR (12.5 µg/mL), VCR (12.5 µg/mL) for additional 24 hours. Apoptosis was analyzed by measuring positive percentage of Annexin V cells via flow cytometry (**C**; n = 3;^ *^ *P*<0.05); cleaved PARP was analyzed by Western blotting (**D**). (**E**) HL60/ADR and K562/A02 cells were transfected with control shRNA or S100A8 shRNA for 48 hours, and then treated with ADR (12.5 µg/mL), VCR (12.5 µg/mL) for additional 24 hours with or without ZVAD-FMK (20 µmol/L). Activation of caspase-3 was analyzed (n = 3;^ *^ *P*<0.05). (**F**) HL60/ADR cells were transfected with control shRNA or S100A8 shRNA (from Gene Pharma, China) for 48 hours and then treated with ADR (12.5 µg/mL), VCR (12.5 µg/mL) for 24 hours. S100A8 protein was determined by Western blot; Cell viability was analyzed by MTT; apoptosis was analyzed by flow cytometry (n = 3;^ *^ *P*<0.05).

### Overexpression of S100A8 increases the resistance of leukemia cells to chemotherapy

To further determine the role of S100A8 in leukemia cells after chemotherapy, we transfected K562 leukemia cells with a plasmid containing full-length human S100A8 cDNA (Fig. 3A). Ectopic overexpression of S100A8 in K562 cells promoted resistance to apoptosis induced by adriamycin and vincristine (Fig. 3B). Autophagy and apoptosis can be triggered simultaneously by common upstream signals [18]. During autophagy, microtubule-associated protein light chain 3 (LC3) is processed post-translationally into soluble LC3-I, and subsequently converted to membrane-bound LC3-II, a marker for autophagosome [19]. Overexpression of S100A8 increased LC3-II following treatment with either ADR or VCR in K562 cells (Fig. 3C). Meanwhile, BECN1, which is necessary for the formation of autophagosomes during the autophagic sequestration process [20], was significantly increased in S100A8 expressing leukemia cells treated with adriamycin or vincristine for 24 h compared with the untreated and control groups (Fig. 3C,D). The polyubiquitin-binding protein SQSTM1/aequestosome 1 (p62) has LC3 binding domains, which target p62 for incorporation into the autophagosomes, thus serving as a selective substrate of autophagy [21]. We found that overexpression of S100A8 increased LC3-II but decreased p62, indicating that p62 degradation is dependent on S100A8-induced autophagy (Fig. 3D,E). Electron microscopy analysis demonstrated that there was increased number of multiple autophagosome-like vacuoles with double-membrane structures in the S100A8 overexpressing cells compared with that of the control group (Fig. 3F).

**Figure 3:** Overexpression of S100A8 increased the resistance of leukemia cells to chemotherapy. (**A**) K562 cells were transfected with control pLPCX or pLPCX-S100A8 plasmids. Protein level of S100A8 was assayed by Western blot. (**B**) K562 cells transfected with control pLPCX or pLPCX-S100A8 plasmids were treated with ADR (1 µg/mL) or VCR (1 µg/mL) for 24 hours. Apoptosis was analyzed by measuring Annexin V–positive cells with flow cytometry (n = 3;^ *^ *P*<0.05). (**C**) K562 cells were treated as B, LC3-I/II and BECN1 levels were assayed by Western blot analysis. **UT,** untreated group of K562 cells transfected with S100A8 plasmids. **Control,** K562 cells were transfected with control pLPCX plasmids. (**D**) K562 cells were transfected with pLPCX control or pLPCX -S100A8 cDNA for 48 hours and then treated with ADR (1 µg/mL) for 24 hours in the presence or absence of bafilomycin A1 (Baf; 100 nmol/L). The protein levels of LC3 and p62 were assayed by Western blot. (**E**) K562 cells were transfected pLPCX or pLPCX-S100A8 cDNA with or without the indicated shRNA for 48 hours. Protein levels of S100A8, PI3KC3, BECN1, Atg7, LC3, and p62 were assayed by Western blots. (**F**) K562 cells transfected with control pLPCX or pLPCX-S100A8 cDNA were subjected to TEM analysis. Autophagosomes were highlighted by arrows. (**G**) K562 cells transfected with PLPCX-S100A8 cDNA were treated with bafilomycin A1 (Baf; 100 nmol/L) or 3-methyladenine (3-MA; 10 mmo/L) for 12 hours. LC3 were assayed by Western blot. **Control,** K562 cells were transfected with control pLPCX. (**H**) K562 cells transfected the indicated shRNA were treated with ADR (1 µg/mL) and VCR (1 µg/mL) for 24 hours. Cell viability was analyzed by MTT assay (n = 3;^ *^ *P*<0.05). NS, not significant.

We further found that increase of S100A8 during anticancer therapy could induce autophagic flux in leukaemia cells. Accumulation of LC3-II was observed in the presence of bafilomycin A1 (an inhibitor of late phase autophagy) in k562 cells both before and after treatment with adriamycin for 24 h compared with the absence of bafilomycin A1 (Fig. 3D). At the same time, overexpression of S100A8 induced autophagic p62 degradation (Fig. 3D).

Bafilomycin A1 increased the induction of LC3-II by S100A8 (Fig 3D), whereas 3-methyladenine, an inhibitor of early-phase autophagy [19], inhibited S100A8-induced LC3-II expression (Fig. 3G). PI3KC3, BECN1 (the mammalian ortholog of yeast Vps30/Atg6), and ATG7 are key regulators of the classical autophagy pathway in mammalian cells [22]. To extend our observation that S100A8 promotes anticancer drug resistance by enhancing autophagy, we knocked down PI3KC3, BECN 1, and Atg7 by shRNA and found that silencing of these genes inhibited LC3-II formation and prevented autophagic p62 degradation in S100A8 overexpressing K562 cells (Fig. 3E). Moreover, downregulation of these genes reversed S100A8-induced protection against chemotherapy (Fig. 3H). These findings indicate that autophagy is required for S100A8-mediated resistance to anticancer agents.

### S100A8 regulates autophagy during chemotherapy in leukemia cells

S100A8 is required for the initiation of As2O3-reduced autophagy in leukemia cells [14]. To further explore the mechanism by which S100A8 regulates autophagy in leukemia cells, we detected LC3-I to LC3-II conversion by immunoblot analysis and LC3 puncta formation by fluorescent imaging analysis. Knockdown of S100A8 inhibited ADR-induced LC3-II (Fig. 4A). LC3 is lipidated and recruited to the autophagosomal membrane following autophagosome formation. Accordingly, accumulation of LC3-II was observed in the presence of bafilomycin A1 (Fig. 4A). Moreover, knockdown of S100A8 inhibited the accumulation of LC3 puncta in leukemia cells as detected by immunofluorenscence with a LC3 antibody (Fig. 4B). In addition, ultrastructural analysis revealed that cells transfected with S100A8 shRNA exhibited fewer autophagosomes during chemotherapy compared with cells transfected with control shRNA (Fig. 4C). To test whether S100A8 influences autophagic flux, we evaluated the expression of p62. Indeed, knockdown of S100A8 inhibited autophagic p62 degradation (Fig. 4A). These findings further support a critical role for S100A8 in the regulation of autophagy in leukemia cells.

**Figure 4:** S100A8 regulated the chemotherapy–induced autophagy in leukemia cells. (**A and B)** K562 cells were transfected with control shRNA or S100A8 shRNA for 48 hours and then treated with ADR (1 µg/mL) and VCR (1 µg/mL) for 24 hours in the presence or absence of bafilomycin A1 (Baf; 100 nmol/L). The protein levels of LC3 and p62 were assayed by Western blot (**A**); LC3 puncta were analyzed by LC3 antibody or mRFP–GFP–LC3 (Magnification is 10×60 oil) (**B**) (n = 3;^ *^ *P*<0.05). (**C**) K562 cells were transfected with control shRNA or S100A8 shRNA for 48 hours and then treated with ADR (1 µg/mL) and VCR (1 µg/mL) for 24 hours. Autophagosome-like structures (indicated by the red arrows) were assayed by TEM (n = 3;^ *^ *P*<0.05). Bar = 2 µm. (**D and E**) K562/A02 cells were transfected with control shRNA or S100A8 shRNA for 48 hours. After pretreatment with rapamycin (Rap; 100 nmol/L) for 6 hours, cells were treated with ADR (1 µg/mL) for 24 hours. Apoptosis was analyzed by measuring Annexin V–positive cells with flow cytometry (**D**). Autophagy was analyzed by measuring LC3 puncta formation (**E**; n = 3;^ *^ *P*<0.05).

Rapamycin induces autophagy by inhibiting the mammalian target of rapamycin complex 1 (mTORC1) [23]. Rapamycin pretreatment prevented ADR from inducing apoptosis in K562/A02 cells (Fig. 4D). However, rapamycin conferred less protection in K562/A02 cells transfected with S100A8 shRNA probably due to diminished autophagic capacity (Fig. 4E). These results suggest that S100A8 is an important regulator of autophagy-mediated leukemia cell survival.

### S100A8 regulates the formation of BECN1–PI3KC3 complex but not ULK1–mAtg13 complex

Mammalian autophagy is a multi-step process including initiation, nucleation, elongation, closure, maturation, and finally degradation or extrusion, and regulated by a core family of ATG proteins [1], [24]. To explore the underlying molecular mechanism of S100A8-mediated autophagy, we analyzed the early autophagic signaling event of ULK1 complex formation. ULK1 is essential for autophagy induction and is comprised of a large complex that includes a mammalian homologue of Atg13 (mAtg13). Knockdown of S100A8 did not affect the formation of ULK1-mAtg13 complex and phosphorylation of ULK1 at Ser55 following ADR treatment (Fig. 5A). However, S100A8 knockdown significantly reduced the formation of the BECN1-PI3KC3 complex (Fig. 5B), which mediates vesicle nucleation during autophagy. Consistent with the previous studies [14], S100A8 formed a complex with BECN1 in leukemia cells (Fig. 5C). Moreover, knockdown of ULK1 inhibited the interaction between S100A8 and BECN1 (Fig. 5C) and potentiated anticancer agent-induced cell apoptosis (Fig. 5D). These data suggest that S100A8 is a downstream signaling molecule from the ULK1-mAtg13 complex and facilitates autophagy in leukemia cells by interacting with BECN1.

**Figure 5:** ULK1-mAtg13 regulated the fomation of S100A8-BECN1 complex formation in leukemia cells. (**A-C**) K562 cells were transfected with S100A8 shRNA (A and B) or ULK1 shRNA (C) for 48 hours and then were treated with ADR (1 µg/mL) for 24 hours. Cells were then processed for immunoprecipitation (IP) or Western blotting (IB) as described in Materials and Methods. All data are representative of 3 experiments. (**D**) K562 cells transfected with S100A8 shRNA (A and B) or ULK1 shRNA (C) for 48 hours were treated with ADR (1 µg/mL) or VCR (1 µg/mL) for 24 hours. Apoptosis was analyzed by measuring Annexin V–positive cells with flow cytometry (n = 3;^ *^ *P*<0.05).

#### RAGE was involved in exogenous S100A8-induced autophagy

To investigate whether extracellular S100A8 induce autophagy in leukemia cells, we treated K562 cells with 1 µg/ml S100A8 protein for 24 h and detected LC3-I/LC3-II and P62 by immunoblot analysis. We found that S100A8 treatment increased the expression of LC3-II, and decreased the expression of p62. To test the role of RAGE and TLR4 in S100A8-induced autophagy, we knocked down RAGE and TLR4 by shRNA in K562 cells. We found that silencing RAGE inhibited LC3-II formation and prevented autophagic p62 degradation. In contrast, knock down of TLR4 did not influence S100A8-induced autophagic flux. These findings indicate that RAGE is involved in exogenous S100A8-induced autophagy (Fig. 6)

**Figure 6:** Exogenous S100A8 regulate autophagy through RAGE receptor. K562 cells were transfected with control shRNA, RAGE shRNA or TLR4 shRNA for 48 hours, and then treated with S100A8 protein (1 µg/ml) for 24 hours. LC3, p62, RAGE and TLR4 were assayed by Western blot. All data were representatives of 3 independent experiments.

## Discussion

Chemotherapy is the major treatment strategy for nearly all types of childhood leukemia [25], [26]; however, drug resistance often renders chemotherapy ineffective and negatively impacts long-term event-free survival [27]. Multidrug resistance results from multiple mechanisms including dysfunctional membrane transport, resistance to apoptosis, and the persistence of stem cell-like leukemia cells. Thus, attenuating drug resistance is a current challenge for the treatment of leukemia.

S100A8 is expressed in a wide variety of cell types and abundant in myeloid cells. Elevated expression of S100A8 has been found in disorders including rheumatoid arthritis, inflammatory bowel disease, and vasculitis [28]. S100A8 and HMGB1 are the ligands of receptor for advanced glycation endproducts (RAGE). RAGE/RAGE ligand interaction is associated with survival of cells expressing this receptor, and is involved in the development and progression of cancer [29]. Inhibition of RAGE interaction with S100p enhanced the anti-tumor activity of conventional chemotherapy in a xenograft model of pancreatic cancer [30]. We previously found that HMGB1-induced autophagy enhances chemotherapy resistance in leukemia cells [16]. It was reported that S100A8 protein balances tumor cell growth and apoptosis in a concentration-dependent manner [31]. Furthermore, variation of S100A8 transcripts has been found in AMLs and correlates with the FAB (French-American-British classification) subtype, or the differentiation of AML [32]. Nevertheless, the role of S100A8 in the pathogenesis of leukemia is unknown.

A number of anticancer therapies, including DNA-damaging chemotherapeutic drugs, induce the accumulation of autophagosomes in tumor cell lines, while pharmacologic inhibition of autophagy or genetic knockdown of phylogenetically conserved autophagy-related genes, such as Atg5 and Atg7, enhanced drug-induced cytotoxicities [33]. The ability to affect chemotherapy sensitivity by regulating autophagy in leukemia cells is a novel function of S100A8 [14]. In this study, we showed that A100A8-mediated autophagy is a significant contributor to drug resistance in leukemia. We found that S100A8 level was elevated in drug resistance leukemia cells relative to the nondrug resistant cells, and vincristine, adriamycin and arsenic trioxide enhanced the expression of S100A8 in human leukemia cells. Further, inhibition of S100A8 or autophagy increased the drug sensitivity of leukemia cells, and knockdown of S100A8 by shRNA increased cell death and suppressed leukemia cell growth. As a member of DAMPs, S100A8 demonstrate an anti-inflammatory, anti-oxidative, and protective effect on cells [34], [35]. The expression of S100A8 in AML patients is associated with worse prognosis and a predictor of poor survival [12]. Thus, it is intriguing to propose that release of S100A8 by dying leukemia cells may help process and present leukemia antigens to immune effector cells.

Cancer cells respond to chemotherapy in a variety of ways, ranging from the activation of survival pathways to the initiation of cell death. Increased autophagy is observed in leukemia cells when exposed to chemotherapy drugs [5], [36]. In general, autophagy is a "programmed cell survival" mechanism to prevent the accumulation of damaged or unnecessary components, but also functions to facilitate the recycling of these components to sustain homoeostasis. Therefore, autophagy functions as a double-edged sword in cancer development and progression by inducing both tumor cell survival and death. In tumor cells, the role of autophagy may depend on the type of tumors and the stage of tumorigenesis [37]. We found that inhibition of autophagy increases leukemia cell death and reverses S100A8-mediated drug resistance. A systematic study on cells exposed to many compounds showed that no single cytotoxic agent can induce cell death by autophagy [38], supporting the observation that autophagy is mostly a cytoprotective mechanism. Here, we found that knockdown of S100A8 decreased LC3 II formation and p62 degradation, which was associated with a decreased number of membrane-bound autophagosomes, as detected by TEM in leukemia cells.

We previously found that S100A8 interacts with BECN1 and displaces Bcl-2 [14]. In the current study, we found that the ULK1-mAtg13 complex is required for the interaction between S100A8 and BECN1, which promotes BECN1-PI3KC3 complex formation. However, the assembly of the BECN1 complexes is complicated and seems to differ in a cell- or tissue-dependent manner [39]. AMP-activated protein kinase (AMPK) is a key molecular player in energy homeostasis and important for the activation of ULK1 [40]. Further studies are needed to test whether AMPK or other kinases are involved in regulating the interaction between S100A8 and BECN1. Finally, we and found that exogenous S100A8 regulates autophagy through its receptor, RAGE, but not TLR4.

In conclusion, we showed that chemotherapy-induced S100A8 expression in leukemia cells promoted autophagy, which in turn inhibited apoptosis and increased drug resistance, indicating that S100A8 is an important regulator of autophagy. Moreover, suppression of S100A8 expression significantly increased drug sensitivity of leukemia cells, suggesting that S100A8 may be a novel target for leukemia therapy. (Fig 7).

**Figure 7:** Scheme of S100A8-mediated autophagy promoting drug resistance in leukemia. Leukemia is the most common type of cancer occurs in childhood. Vincristine and adriamycin are the commonly used cytotoxic anticancer drugs in the treatment of patients with Leukemia. These drugs increase endogenous mRNA and protein expression of S100A8 in Leukemia cells by an unknown mechanism. Upregulated S100A8 competes with BCL-2 to bind BECN1, which increases the formation of the BECN1-PtdIns3KC3 complex and stimulates autophagosome maturation and autophagy. As an upstream signal, activation of the ULK1-mATG13 complex is required for the interaction between S100A8 and BECN1. Knockdown of S100A8 or inhibition of autophagy increase apoptosis, and reverses drug resistance in leukemia cells. Furthermore, exogenous S100A8 regulates autophagy through the RAGE receptor. Thus S100A8-mediated autophagy is a potential therapeutic target for leukemia.
